This article has been retracted.

# Analysis of Multigene Mutations in Lung Adenocarcinoma in Zunyi

**DOI:** 10.1155/2021/9939065

**Published:** 2021-05-28

**Authors:** Qingqing Ma, Dengming Ma, Mu Lin, Yadong Gong, Xiaojing Han, Yunhua Chen, Zhu Tang, Mubo Liu

**Affiliations:** ^1^Department of Central Laboratory, Guizhou Aerospace Hospital, Guizhou 563000, China; ^2^Department of Anesthesiology, First People's Hospital of Mengyin County, China

## Abstract

**Objective:**

Driver gene mutation in lung adenocarcinoma patients in Zunyi and its relationship with clinical features were probed in this investigation.

**Methods:**

In total, with 244 patients with lung adenocarcinoma as study subjects, including 141 males and 103 females, amplification-refractory mutation system-polymerase chain reaction (ARMS-PCR) was utilized for detecting multigene mutations. Subsequently, the relationship between gene mutation and clinical characteristics was analyzed.

**Results:**

The total mutation rate of driver genes was 65.17%, including 48.36% EGFR, 6.15% KRAS, 5.74% ALK, 2.05% HER-2, 1.23% ROS1, 0.82% RET, 0.41% NRAS, and 0.41% BRAF. Among EGFR mutations, 47.46% were EGFR-19-deletion, 42.37% EGFR-21-L858R mutation, 4.24% EGFR-20-T790M mutation, 2.54% EGFR-21-L861Q mutation, 2.54% EGFR-20-insertion, and 0.85% EGFR-18-G719X mutation. Both female patients and nonsmoking patients with lung adenocarcinoma had a higher rate of EGFR mutation. Additionally, 15 patients with multiple mutations in EGFR, including 13 patients with 2 mutations in EGFR and 2 patients with 3 mutations in EGFR, were found.

**Conclusion:**

Among driver gene mutations in patients with lung adenocarcinoma in Zunyi, EGFR mutation has the highest incidence, followed by ALK fusion and KRAS mutation. Although both mutations and multisite mutations in the other driver genes account for a low proportion, they still have great clinical significance. Multigene mutation detection contributes to the rapid screening of patients with lung adenocarcinoma who respond to targeted therapy.

## 1. Introduction

Lung cancer is a common malignant tumor associated with the highest prevalence and mortality in China [1]. Non-small cell lung cancer (NSCLC) and small cell lung cancer are its main subtypes, the former accounting for about 85% of lung cancer and the latter approximately 15%. Lung adenocarcinoma contributes the most to the NSCLC, accounting for almost 50% of lung cancer [2]. At present, the commonly employed treatment for lung adenocarcinoma includes surgery in the early stage and chemotherapy in the late stage. However, due to insufficient awareness of screening and backward diagnostic techniques, most patients are diagnosed when they reach an advanced stage, thus resulting in lower overall survival. Therefore, the study on lung adenocarcinoma-related genes and signaling pathways is meaningful work, which contributes to the improvement of molecular diagnosis and molecular therapy for early lung adenocarcinoma [3].

Numerous clinical studies have shown that driver gene mutation can be served as a predictor of the efficacy of targeted drugs. For example, a series of driver gene mutations such as epidermal growth factor receptor (EGFR) gene mutation, anaplastic lymphoma kinase (ALK) fusion, or receptor tyrosine kinase (ROS1) fusion significantly affect the development of lung adenocarcinoma [4]. With the development of molecular diagnostics technology, the discovery of lung cancer driver genes like EGFR, Kirsten rat sarcoma 2 viral oncogene homolog (KRAS), ALK, and ROS1 has laid the foundation for genotyping, individualized treatment, and targeted therapy [5].

In NSCLC patients in China, the positive rate of EGFR mutation is 40%-50%, followed by KRAS (15%-30%), ALK (3%-7%), ROS1 (1%-2%), and RET protooncogene (RET) (1%-2%) [6]. In 2020, the Chinese Society of Oncology (CSCO) clearly indicated that regardless of their clinical characteristics (such as smoking history, gender, ethnicity, or others), all NSCLC patients with adenocarcinoma should be routinely tested for EGFR mutation, ALK fusion, and ROS1 fusion, and the detection of EGFR mutation should include exons 18, 19, 20, and 21 of the EGFR gene [7]. Studies have shown that only some patients are sensitive to EGFR tyrosine kinase inhibitors (EGFR-TKIs), such as gefitinib and erlotinib. However, the presence of mutation in EGFR exons 18-21 can lead to a stronger response of EGFR to epidermal growth factor and increased tyrosine kinase activity, thus resulting in enhanced sensitivity to EGFR-TKIs and better efficacy [8]. Collectively, the detection of driver genes, especially the multigene detection, and the analysis of gene mutations are of great significance for the treatment of patients with lung cancer.

At present, the commonly used technologies for multigene detection mainly include amplification-refractory mutation system-polymerase chain reaction (ARMS-PCR) and next-generation sequencing (NGS) [9]. ARMS-PCR can simultaneously determine multiple specified genes, with low requirements for DNA concentration and quality of the samples, high sensitivity, convenient and quick operation, and high efficiency [10]. This method is feasible for the detection of all 8 core driver genes EGFR, ALK, ROS1, NRAS, RET, KRAS, BRAF, and HER-2 genes recommended by the latest version of the National Comprehensive Cancer Network (NCCN) guidelines [11]. Increasing small-molecule inhibitors are utilized in clinical practice, and their efficacy and drug resistance mechanism are closely related to gene mutations. Therefore, genetic testing contributes to the determination of a specific treatment plan. Notably, the significant differences in EGFR gene mutations in patients with lung cancer in different regions is supported by some reports, but few studies on the genetic testing for patients with lung adenocarcinoma in Zunyi [12]. Therefore, in this paper, paraffin-embedded tissue sections obtained from 244 patients with lung adenocarcinoma in Zunyi, Guizhou province, were detected by ARMS-PCR. Based on the detection, we aimed to analyze the correlation between driver gene mutation and clinicopathologic features, thus providing a reference for better diagnosis and treatment of lung cancer patients.

## 2. Materials and Methods

### 2.1. Clinical Data

In total, 244 patients (141 males and 103 females, mean age: 63.03 ± 10.82 years) diagnosed with lung adenocarcinoma by pathological and cytological examination, who were admitted to Guizhou Aerospace Hospital between May 2015 and December 2020, were included. On completion of the fixation step by formaldehyde, the pathological tissue samples were embedded in paraffin, then sectioned and finally stained with HE. A professional pathologist determined the pathological type and number of tumor cells. Subsequently, ARMS-PCR was utilized for detecting mutations of 10 driver genes.

### 2.2. Reagents and Instruments

The main experimental instruments included the SLAN-96 PCR system (ABI, USA), ultramicro spectrophotometer, FFPE DNA/RNA nucleic acid extraction kit (FFPE RNA), and ten human gene mutation (EGFR, ALK, ROS1, RET, KRAS, MRAS, BRAF, HER-2, PIK3CA, and MET) fluorescence PCR diagnostic kits. The above two kits were provided by AmoyDx, China. The experimental operation was carried out in strict accordance with the instructions of instruments and kits.

### 2.3. DNA Extraction

In total, after being placed in a 1.5 mL EP tube, 10-20 sections of paraffin-embedded tissues with at least 200 tumor cells were utilized for DNA and RNA extraction by FFPE DNA/RNA nucleic acid extraction kit. The specific steps were as follows: (1) xylene for deparaffinization, (2) absolute ethanol for elution, (3) proteinase K solution for tissue lysis, and (3) special adsorption columns for extraction of DNA and RNA from the tissues. Measurement of the DNA concentration was conducted by the ultramicro spectrophotometer (1 *μ*g/*μ*L), and the A260/A280 ranged from 1.8 to 2.1.

### 2.4. Gene Mutation Analysis

All gene statuses were assayed by using gene mutation fluorescence PCR diagnostic kits according to the manufacturer's instructions and as previously reported [13]. Extracted genomic DNA was added to the reaction system, and after amplification, fluorescent signals were collected from the 6-carboxyfluorescein (FAM) and hexachlorofluorescein channels. Genotypes were determined based on changes in threshold counts and/or count values as indicated in the manufacturer's instructions.

### 2.5. Statistical Analysis

Statistical analysis of all data was carried out by using SPSS 23.0. Evaluation of the relationship between each gene mutation and NSCLC clinicopathologic features of NSCLC was evaluated by a chi-square test with correction for continuity and Fisher's exact test. A significant difference was suggested if *P* < 0.05.

## 3. Results

### 3.1. Driver Gene Mutations

In 244 patients with lung adenocarcinoma, the total mutation rate of driver genes was 65.17%, including EGFR 48.36% (118/244), KRAS 6.15% (15/244), ALK 5.74% (14/244), HER-2 2.05% (5/244), ROS1 1.23% (3/244), RET 0.82% (2/244), NRAS 0.41% (1/244), BRAF 0.41% (1/244), PIK3CA 0.00% (0/244), and MET 0.00% (0/244). And 34.83% (85/244) of the patients had no detectable mutation (Table 1).

### 3.2. EGFR Gene Mutations

It has been reported that more than 90% of EGFR mutations exist in exons 18-21, and deletion mutation in exon 19 (EGFR-19-Del) and L858R missense mutation in exon 21 (EGFR-2-L858R) are the most common. In our results (Table 2), the overall mutation rate of the EGFR gene in patients with lung adenocarcinoma was 48.36%, including 47.46% (56/118) EGFR-19-Del, 42.37% (50/118) EGFR-21-L858R, 4.24% (5/118) EGFR-20-T790M mutation, 2.54% (3/118) EGFR-21-L861Q mutation, 2.54% (3/118) EGFR 20-insertion, and 0.85% (1/118) EGFR-18-G719X mutation.

### 3.3. Multiple Mutations in EGFR

In total, 15 patients with multiple mutations in EGFR were found in this study, including 13 patients with 2 mutations in EGFR and 2 patients with 3 mutations in EGFR. Among the mutations, EGFR-19-Del combined with EGFR-20-T790M mutation accounted for the highest proportion, 2.87% (7/15) (Table 3). For the clinical information of patients with multiple mutations in EGFR, see Table 4.

### 3.4. Relationship between EGFR Gene Mutations and Clinical Characteristics

As shown in Table 5, among all the patients, female patients and patients in Han regions were more likely to have driver gene mutations (*P* < 0.05). Further analysis revealed that the patients with an age ≥ 63 and no smoking history were more prone to EGFR mutations (*P* < 0.05), but there were no significant differences in nation and lymph node metastasis.

## 4. Discussion

According to the latest global cancer data released in February 2020, there were 24.5 million new cancer cases and 9.6 million cancer-caused deaths worldwide in 2017. Among the malignant tumors reported, the global incidence and mortality of lung cancer rank second and first, respectively, while its incidence ranks first in China [14]. Clinically, surgery, chemotherapy, and radiotherapy are mainly utilized for lung cancer. However, although these traditional treatments have been greatly improved, the overall efficacy and prognosis are still poor, and the survival rate is low [15]. Molecular targeted therapy, in recent years, has been rapidly developed and widely used due to its safety, effectiveness, and simplicity. EGFR, ALK, and KRAS are relatively common and well-studied driver genes in lung adenocarcinoma, which are not only involved in the development of lung adenocarcinoma but also related to the resistance to small molecule targeted inhibitors. Therefore, driver gene detection in patients with lung adenocarcinoma can serve as a guide for molecular targeted therapy and contributes to the research and development of antiresistance inhibitors.

EGFR is a transmembrane receptor widely distributed in mammalian epithelial cells, fibroblasts, and other cells, indicating the correlation of the EGFR signaling pathway with proliferation and metastasis, angiogenesis, and apoptosis of tumor cells. In patients with lung adenocarcinoma, common EGFR mutations mainly include 4 types: point mutation in exon 18, deletion in exon 19, insertion in exon 20, and point mutation in exon 21 [8]. Approximately 90% of these four types are EGFR-19-Del and EGFR-2-L858R, and these two also accounted for 89.83% of EGFR mutations in this study. EGFR-19-Del mostly occurs at amino acids 746 to 750, which can change the ATP-binding poke angle, and further enhance the sensitivity of tumor cells to small-molecule TKIs. EGFR-2-L858R is characterized by a leucine to arginine mutation at codon 858. Clinical studies have also shown that these two mutants have significant biological characteristics and can affect the response to EGFR-TKIs. Not all patients can benefit from EGFR-TKIs; females, nonsmokers, adenocarcinoma patients, and East Asian populations benefit most from EGFR-TKIs [16]. Collectively, therefore, detection of gene mutations in patients with lung adenocarcinoma is of significance for the selection of targeted therapeutic drugs. In this paper, we found that although multiple mutations in EGFR had low incidence (6.15%, 15/244), they are still of vital importance to targeted and individualized treatment.

Significant differences in EGFR mutations in patients with lung adenocarcinoma in different regions of China are supported by literature [17]. As reported, in lung adenocarcinoma patients in China, the mutation rate of EGFR gene was 59.04% in Jiaxing [18], 48.7% in Shenzhen [19], 48.9% in Chongqing [20], 52.8% in Hangzhou [21], 47.15% in southern Anhui [22], and 41.04% in Shandong [23]. We revealed that the total mutation rate of 10 common driver genes in patients with lung adenocarcinoma in Zunyi was 71.72%, which was consistent with a previous report by Huang et al. [24]. Additionally, among the mutations of these 10 driver genes, EGFR mutation had the highest proportion, accounting for 48.36%, which was consistent with the result of Sui et al. [25]. Further analysis of mutation sites showed that EGFR-19-Del (22.95%, 56/244) and EGFR-21-L858R (20.49%, 50/244) were the main types of EGFR mutations in patients with lung adenocarcinoma in Zunyi. Collectively, EGFR mutations are not the same in patients with lung adenocarcinoma in different regions. It is also possible that this is related to the influence of multiple factors such as different living environments of people in different regions, different dietary habits, and different sample inclusion sizes, which make a large difference between the results of domestic studies on EGFR gene mutations in NSCLC [26, 27]. Therefore, detection of gene mutation is of vital importance for guiding personalized and targeted medication.

In addition to EGFR, other driver genes like KRAS, ALK, and ROS1 have value in guiding clinical medication for patients with lung adenocarcinoma. To this end, investigation of the specific mutation rate of these driver genes was also carried out. KRAS gene mutation was 6.15% (15/244), consistent with the mutation rate of 4%-24% in the Asian population. ALK fusion rate was 5.74% (14/244), followed by HER-2 gene mutation (2.05%, 5/244), ROS1 gene mutation (1.23%, 3/244), RET gene mutation (0.82%, 2/244), NRAS gene mutation (0.41%, 1/244), and BRAF gene mutation (0.41%,1/244). Although the latter 5 gene mutations are rare mutations with low incidence, the choice of treatment remains crucial for patients with positive mutations of these driver genes.

It is reported in the existing literature that the incidence of EGFR mutation is higher in Asian nonsmoking females with lung adenocarcinoma; KRAS mutation is associated with smoking, which is more common in male patients with lung adenocarcinoma; and ALK and ROS1 fusion mutations have higher frequency in nonsmoking young patients. Consistent results were obtained by our study with the previous literature in determination of the relationship between EGFR mutation and clinicopathologic features. But we found no significant relationship between the other driver gene mutations, which are rare, and clinicopathologic features, probably because of the number of cases included. Multigene mutations can occur in patients with lung cancer, such as EGFR mutation combined with ALK fusion [24]. However, in this study, only patients with multiple mutations in EGFR but not patients with multigene mutations were found, which may be related to the number of samples.

## 5. Conclusion

In summary, there is a high mutation rate of the EGFR gene in lung adenocarcinoma. Although multiple mutations in other driver genes and multigene mutations account for a low proportion, they still have great significance for clinical targeted and individualized treatment. Therefore, combined detection of gene mutation is recommended for an initial treatment for lung cancer patients or population screening. In addition to surgery, chemoradiotherapy, and immunotherapy, this detection contributes to the rapid screening of patients with lung adenocarcinoma who respond to targeted therapy, which can improve the efficacy, maximize the quality of life, and prolong the survival of patients.

## Figures and Tables

**Table 1:** Driver gene mutations.

Mutant gene	Gender	Mutation rate (%, *n* = 244)
EGFR	M = 59, F = 59	118 (48.36)
KRAS	M = 8, F = 7	15 (6.15)
ALK	M = 3, F = 11	14 (5.74)
HER-2	M = 4, F = 1	5 (2.05)
ROS1	M = 2, F = 1	3 (1.23)
RET	M = 1, F = 1	2 (0.82)
NRAS	M = 1, F = 0	1 (0.41)
BRAF	M = 0, F = 1	1 (0.41)
PIK3CA	M = 0, F = 0	0 (0.00)
MET	M = 0, F = 0	0 (0.00)
Not detect	M = 63, F = 22	85 (34.84)

**Table 2:** EGFR gene mutation.

Mutant gene	Gender	Mutation rate (%, *n* = 244)	Percentage/EGFR mutation (%, *n* = 118)
EGFR-19-deletion	M = 26, F = 30	56 (22.95)	56 (47.46)
EGFR-21-L858R mutation	M = 24, F = 26	50 (20.49)	50 (42.37)
EGFR-20-T790M mutation	M = 4, F = 1	5 (2.05)	5 (4.24)
EGFR-20-insertion	M = 2, F = 1	3 (1.23)	3 (2.54)
EGFR-21-L861Q mutation	M = 2, F = 1	3 (1.23)	3 (2.54)
EGFR-18-G719X mutation	M = 1, F = 0	1 (0.41)	1 (0.85)

**Table 3:** Multiple mutations in EGFR.

Mutant gene	Gender	Mutation rate (%)
Del+T790M	M = 2, F = 5	7 (2.87)
T790M+L858R	M = 1, F = 1	2 (0.82)
G719X+S768I	M = 2, F = 0	2 (0.82)
G719X+L858R	M = 0, F = 1	1 (0.41)
G719X+T790M	M = 0, F = 1	1 (0.41)
Del+G719X+S768I	M = 0, F = 1	1 (0.41)
Del+T790M+L858R	M = 1, F = 0	1 (0.41)

**Table 4:** Clinical information of 15 patients with multiple mutations in EGFR.

	Gender	Age	Pathological type	Smoking history	Mutation type
Case 1	Female	44	Adenocarcinoma	No	Del+T790M
Case 2	Female	47	Adenocarcinoma	No	G719X+T790M
Case 3	Male	47	Adenocarcinoma	Yes	T790M+L858R
Case 4	Male	51	Adenocarcinoma	Yes	Del+T790M
Case 5	Female	51	Adenocarcinoma	No	Del+T790M
Case 6	Female	57	Adenocarcinoma	No	G719X+L858R
Case 7	Female	57	Adenocarcinoma	No	Del+T790M
Case 8	Male	58	Adenocarcinoma	Yes	G719X+S768I
Case 9	Female	59	Adenocarcinoma	No	Del+T790M
Case 10	Female	63	Adenocarcinoma	No	Del+G719X+S768I
Case 11	Male	67	Adenocarcinoma	Yes	Del+T790M
Case 12	Male	69	Adenocarcinoma	No	Del+T790M+L858R
Case 13	Female	70	Adenocarcinoma	No	T790M+L858R
Case 14	Female	76	Adenocarcinoma	No	Del+T790M
Case 15	Male	76	Adenocarcinoma	Yes	G719X+S768I

**Table 5:** Relationship between gene mutations and clinical characteristics in patients with lung adenocarcinoma.

Clinical pathology parameter	Driver gene		*P*	EGFR mutation	Other gene mutations	*P*
	Mutation	No mutation				
Gender						
Male	84 (34.43)	57 (23.36)	0.001	65 (26.64)	19 (7.79)	0.808
Female	91 (37.30)	12 (4.92)		69 (28.28)	22 (9.02)	
Age						
<63	75 (30.74)	30 (12.30)	0.930	52 (21.31)	23 (9.43)	0.050
≥63	100 (40.98)	39 (15.98)		82 (33.61)	18 (7.38)	
Nation						
Han	127 (52.05)	78 (31.97)	0.033	77 (31.56)	50 (20.49)	0.544
Other	17 (6.97)	22 (9.02)		9 (3.69)	8 (3.28)	
Smoking history						
Yes	55 (22.54)	21 (8.61)	0.755	27 (11.07)	28 (11.48)	0.009
No	119 (48.77)	50 (20.49)		83 (34.02)	36 (14.75)	
Lymph node metastasis						
Yes	52 (21.31)	22 (9.02)	0.822	36 (14.75)	16 (6.56)	0.911
No	117 (47.95)	53 (21.72)		82 (33.61)	35 (14.34)	

## Data Availability

All data are available in this paper.

## References

[1] Liu X., Cho W. C. (2017). Precision medicine in immune checkpoint blockade therapy for non-small cell lung cancer. *Clinical and Translational Medicine*.

[2] Sun G. Z., Zhao T. W. (2019). Lung adenocarcinoma pathology stages related gene identification. *Mathematical Biosciences and Engineering*.

[3] Siegelin M. D., Borczuk A. C. (2014). Epidermal growth factor receptor mutations in lung adenocarcinoma. *Laboratory Investigation*.

[4] Oberndorfer F., Müllauer L. (2018). Molecular pathology of lung cancer: current status and perspectives. *Current Opinion in Oncology*.

[5] Duma N., Santana-Davila R., Molina J. R. (2019). Non-small cell lung cancer: epidemiology, screening, diagnosis, and treatment. *Mayo Clinic Proceedings*.

[6] Wang Y., Yu L., Fang N., Sun B. (2019). Genetic mutations among Chinese patients with non-small cell lung cancer and targeted therapy. *Zhonghua yi xue yi chuan xue za zhi= Zhonghua yixue yichuanxue zazhi= Chinese journal of medical genetics*.

[7] (2020). Guidelines Of Chinese Society Of Clinical Oncology (CSCO), Non-Small Cell Lung Cancer 2020.

[8] Lynch T. J., Bell D. W., Sordella R. (2004). Activating mutations in the epidermal growth factor receptor underlying responsiveness of non-small-cell lung cancer to gefitinib. *The New England Journal of Medicine*.

[9] Wang Z., Chen R., Wang S. (2014). Quantification and dynamic monitoring of EGFR T790M in plasma cell-free DNA by digital PCR for prognosis of EGFR-TKI treatment in advanced NSCLC. *PLoS One*.

[10] Ellison G., Donald E., McWalter G. (2010). A comparison of ARMS and DNA sequencing for mutation analysis in clinical biopsy samples. *Journal of Experimental & Clinical Cancer Research*.

[11] Ning Y., Xie D., She Y. L. (2020). An interpretation of the NCCN guideline for lung cancer screening: 2020 version. *Chinese Journal of Clinical Thoracic and Cardiovascular Surgery*.

[12] Yang C. S., Xu W. M., Feng Q., Wang Y. Y., Pan X. Y., Wang L. (2016). EGFR gene mutation of non-small cell lung cancer from different regions of Yunnan province. *Medical Journal of National Defending Forces in Southwest China*.

[13] Wan R., Wang Z., Lee J. J. (2017). Comprehensive analysis of the discordance of EGFR mutation status between tumor tissues and matched circulating tumor DNA in advanced non-small cell lung cancer. *Journal of Thoracic Oncology*.

[14] Yabo S. (2018). National cancer statistics 2018. *China Medical Information Herald*.

[15] Fang M. Y., Wang S. Y., Zheng Y. B. (2014). Prognostic and predictive significance of plasma hepatocyte growth factor and carcinoembryonic antigen in non-small lung cancer after surgery. *European Review for Medical and Pharmacological Sciences*.

[16] Pao W., Miller V., Zakowski M. (2004). EGF receptor gene mutations are common in lung cancers from "never smokers" and are associated with sensitivity of tumors to gefitinib and erlotinib. *Proceedings of the National Academy of Sciences*.

[17] Chen Y. J., Roumeliotis T. I., Chang Y. H. (2020). Proteogenomics of non-smoking lung cancer in East Asia delineates molecular signatures of pathogenesis and progression. *Cell*.

[18] Zhang J., Zhang F., Zhou L. (2017). EGFR mutations and clinicopathological features in patients with non-small cell lung cancer. *Zhejiang Medical Journal*.

[19] Wang L. A., Wang L.-f., Liu A.-s., Yu S.-l. (2017). Analysis of EGFR gene mutation in 103 patients with non-small cell lung cancer in Shenzhen. *Journal of Clinical Transfusion and Laboratory Medicine*.

[20] Ge J., Li L., Yao X., Yan X., Bian X., Luo T. (2019). Analysis of EGFR mutation and clinical characteristics in 924 patients with non-small cell lung cancer in Chongqing. *Chinese Journal of Clinical and Experimental Pathology*.

[21] Zhao Z., Zhou Y. L. (2016). Analysis of EGFR,KRAS and BRAF mutations in 89 cases of lung adenocarcinoma in Hangzhou. *Chinese Journal of Health Laboratory Technology*.

[22] Luo Z. F. H. (2016). Analysis of clinical characteristics and mutation of non small cell lung cancer EGFR in the south of Anhui Province. *Journal of Qiqihar University of Medicine*.

[23] Qiao X., Ai D., Liang H., Mu D., Guo Q. (2017). Gene expression and clinical characteristics of molecular targeted therapy in non-small cell lung cancer patients in Shandong. *Chinese Journal of Lung Cancer*.

[24] Huang Q., Chen T., Chen H. (2019). Relationship between driver gene mutation and clinicopathological features in 300 cases of non-small cell lung cancer based on next generation sequencing. *Chinese Journal of Clinical and Experimental Pathology*.

[25] Sui Y., Deng X., Wu Z. (2020). Comprehensive investigation of driver gene expression and clinicopathological characteristics in non-small cell lung cancer. *Journal of Clinical and Experimental Pathology*.

[26] Yang Mei Z. L., Jianqing Z., Bai G., Aili M. (2016). The difference of EGFR mutations in Uyghur and Han's non-small cell lung cancer in Xinjiang, China. *Modern Oncology*.

[27] Gao Y., Li M., Xing S. (2019). Analysis of EGFR gene mutation detection in non-small cell lung cancer patients in Baotou, Inner Mongolia. *Chinese Journal of Clinical Laboratory Science*.

